The article "ResNet-BiLSTM: A Multiscale Deep Learning Model for Heartbeat Detection Using Ballistocardiogram Signals" was retracted in 2023. Reasons: signs of a paper mill; compromised peer review; unreliable results or conclusions.

# ResNet-BiLSTM: A Multiscale Deep Learning Model for Heartbeat Detection Using Ballistocardiogram Signals

**DOI:** 10.1155/2022/6388445

**Published:** 2022-01-27

**Authors:** Yijun Liu, Yifan Lyu, Zhibin He, Yonghao Yang, Jinheng Li, Zhiqiang Pang, Qinghua Zhong, Xuejie Liu, Han Zhang

**Affiliations:** ^1^School of Electronics and Information Engineering, South China Normal University, Guangzhou 510006, China; ^2^Guangzhou SENVIV Technology Co. Ltd, Guangzhou 510006, China; ^3^Guangdong Provincial Engineering Technology Research Center of Cardiovascular Individual Medicine and Big Data, South China Normal University, Guangzhou 510006, China

## Abstract

As the heartbeat detection from ballistocardiogram (BCG) signals using force sensors is interfered by respiratory effort and artifact motion, advanced signal processing algorithms are required to detect the J-peak of each BCG signal so that beat-to-beat interval can be identified. However, existing methods generally rely on rule-based detection of a fixed size, without considering the rhythm features in a large time scale covering multiple BCG signals. *Methods*. This paper develops a deep learning framework based on ResNet and bidirectional long short-term memory (BiLSTM) to conduct beat-to-beat detection of BCG signals. Unlike the existing methods, the proposed network takes multiscale features of BCG signals as the input and, thus, can enjoy the complementary advantages of both morphological features of one BCG signal and rhythm features of multiple BCG signals. Different time scales of multiscale features for the proposed model are validated and analyzed through experiments. *Results.* The BCG signals recorded from 21 healthy subjects are conducted to verify the performance of the proposed heartbeat detection scheme using leave-one-out cross-validation. The impact of different time scales on the detection performance and the performance of the proposed model for different sleep postures are examined. Numerical results demonstrate that the proposed multiscale model performs robust to sleep postures and achieves an averaged absolute error (*E*_abs_) and an averaged relative error (*E*_rel_) of the heartbeat interval relative to the R-R interval of 9.92 ms and 2.67 ms, respectively, which are superior to those of the state-of-the-art detection protocol. *Conclusion.* In this work, a multiscale deep-learning model for heartbeat detection using BCG signals is designed. We demonstrate through the experiment that the detection with multiscale features of BCG signals can provide a superior performance to the existing works. Further study will examine the ultimate performance of the multiscale model in practical scenarios, i.e., detection for patients suffering from cardiovascular disorders with night-sleep monitoring.

## 1. Background

The World Health Organization (WHO) announced that cardiovascular disease (CVD) causes the highest mortality in the world, where approximately 17.1 million people died of CVD every year. Clinical studies have shown that continuous vital sign monitoring (including heart rate and respiratory rate) is of great significance for the early detection of CVD [1–3]. As the gold standard of heart rate monitoring, electrocardiogram (ECG)-based technologies have been widely used over the past several decades. Compared with the ECG, ballistocardiogram (BCG)-aided heart rate monitoring, as a noninvasive, simple operation and low-cost technique, has received extensive attention in the fields of both academia and industry. In pioneer studies [4, 5], the authors developed a noninvasive BCG acquisition system by using force sensors, where heart rate was computed based on the detection of J-peaks from BCG signals. As has been verified by Mack et al. and Kim et al. [6, 7], J-J interval of the BCG signal is highly consistent with the R-R interval of the ECG signal, from which heart rate variability (HRV) can be obtained. Since the acquisition of the BCG signal is contactless with the human body, such a noninvasive heartbeat detection is promising for the application of in-home monitoring. For example, sensors can be integrated into bed [8, 9], chair [10, 11], and pillow [12]. However, the robustness of noninvasive vital sign acquisition in practical scenarios is limited [4], where the reasons can be summarized as twofold. First, for noninvasive sensing, the acquisition of BCG is significantly interfered by the respiratory effort and artifact motion. Second, the morphology of BCG may differ between people of different body weights, gender, and healthy status, which brings challenges to the detection.

For heartbeat detection, most of the conventional schemes of heartbeat detection are based on the criterion of template matching. To be specific, the authors in [13] proposed to extract the envelope of the BCG signal with Hilbert transform and then calculated the averaged heart rate in the frequency domain using the fast Fourier transform. For beat-to-beat detection, the authors in [14, 15] employed discrete wavelet transform and filter banks to extract BCG signals from the mixed vital signs, where the heartbeat interval was obtained by identifying the J-peak of each BCG signal. In [16], Lee et al. proposed to detect the J-peak of the BCG signal in the time domain with Shannon entropy-based nonlinear filtering. As an alternative to J-peak detection of BCG signals, in [17], a heartbeat shape was adaptively modeled based on a two-step procedure by taking advantage of the J-peak and the K-valley of BCG signals. Then, the forward and backward detections with the criteria of both the morphological distance and the cross-correlation were jointly employed to find the position of each BCG signal. Similarly, Bruser et al. [18] proposed to generate the model by using the *K*-means clustering algorithm. To be specific, within each 30 s epoch of BCG signals, *K*-means clustering was applied to generate the maximum likelihood heartbeat model, by which the J-peak of each BCG was identified using second-order statistics. Although the experimental results are promising, it is noted that the modeling-based schemes [17, 18] require prior information of BCG signals. To elaborate, during the interval interfered by respiratory effort and artifact motion, modeling of BCG is challenging since the shape of each BCG signal over an epoch is nonrobust. Moreover, the J-peak detection is based on a sliding window of a fixed time scale, ranging from 0.5 s to 1.5 s [19, 20]. That means, heartbeat detection is infeasible in cases of tachycardia (i.e., heart rate >100 beats/s) or bradycardia (i.e., heart rate <40 beats/s). Specifically, the aforementioned scheme is based on template matching using a sliding window of a fixed time scale (typically ranges from 0.5 to 2 s). That means, errors of heartbeat detection will occur for the cases of either heart rate >120 beats/min or <30 beats/min.

In recent years, deep learning has been widely used in the field of healthcare and achieved great success as Amritphale et al. [21] presented a deep neural network-based artificial intelligence prediction model to help identify a subgroup of patients undergoing carotid artery stenting who are at risk for short-term unplanned readmissions. And in recent studies, deep learning (DL) technologies have been applied for heartbeat detection. In [22], Zhang et al. employed the convolutional neural network (CNN) combined with the extreme learning machine to detect the J-peak of the BCG signal. In [23], Jiao et al. proposed a BCG detection algorithm based on multi-instance and dictionary learning, where the feature dimensions were firstly reduced by dictionary learning, and semisupervised learning method, i.e., multi-instance learning, was then used for classification. To the latest contribution, Hai et al. proposed to use the GRU neural network for BCG detection [20]. Compared with the conventional rule-based detection [13–19], DL-based methods can address the limitation of a fixed-scale decision. Intuitively, the detection of the J-peak depends not only on the details of the current BCG signal but also relies on the priori information of temporal rhythm across adjacent intervals in a large time scale. However, such rhythm features over multiple BCG signals were not considered by the existing DL methods [20, 22, 23].

To address the above issues, we proposed a deep learning-based heartbeat detection scheme, which performs robust to different heart rate conditions. Specifically, the contributions of the proposed heartbeat detection, in comparison with the pioneer studies, are listed as follows:

1. The proposed DL model takes the advantages of both ResNet and BiLSTM, by which the depth-related features, high-level semantic features, and the memory information characterizing the dependency of BCG features in a relatively wide time scale can be extracted.
2. Taking the time-series BCG signals of different scales as the input, multiscale features, i.e., both fine-grained morphological features of each BCG signal (in a small time scale) and rhythm features across multiple BCG signals (in a large time scale), can be fused to improve the detection performance.
3. In the experimental study, 21 subjects with different ages, genders, and measurement postures are considered to validate the effectiveness of the proposed DL model. Compared with the state-of-the-art methods [17, 18, 23], the proposed multiscale DL model yields a superior performance in terms of averaged absolute error and relative error, respectively.

## 2. Methods

### 2.1. Overview

The diagram of the proposed heartbeat detection scheme is shown in Figure 1. Firstly, vital signs are measured in a contactless manner using a piezoelectric sensor. With the data preprocessing, the impacts of respiratory effort and noise on BCG signals are removed, and the resulting BCG signals of different time scales are fed into the proposed ResNet-BiLSTM model for feature extraction and heartbeat identification.

### 2.2. Vital Sign Acquisition

In this paper, BCG is recorded in a noncontact manner by using a noninvasive sensing system (as known as “witheart”), which is developed by Guangzhou Senviv Tech. Co., Ltd., P. R. China (https://www.senviv.com). The system is composed of a piezoelectric sensor unit for vital sign acquisition and a signal processing unit with a sampling frequency of 1 kHz for data processing. It has a 16 bit analog-to-digital converter (ADC) to convert analog signals into digital signals for subsequent processing and analysis. For vital sign acquisition, the sensing unit is placed under the pillow so that BCG and respiratory signals can be recorded simultaneously in a noncontact manner. The scenario of vital sign acquisition is shown in Figure 2.

For reference and comparison, during the noncontact acquisition phase, BIOPAC MP160 physiological recorder is used to record ECG signals with a sampling rate of 1 kHz, simultaneously. Similar to the existing study, ECG signal is regarded as the ground truth for labeling. To be specific, J-peaks of BCG signals are manually synchronized to R-peaks of ECG signals, and the samples within the duration of each BCG signal are labeled as the signal of interest. The manually synchronized BCG and ECG are shown in Figure 3.

In this study, 21 volunteers (17 males and 4 females, aged 22.3 ± 3 years, with averaged heart rate 72 ± 16 bpm, body weight 59.5 ± 16 kg, and height 171.3 ± 8.2 cm) without cardiovascular disease are participated in the experiments. In the process of BCG acquisition, the average duration of vital sign acquisition of each volunteer is longer than 20 minutes, and the total ratios of the supine posture, left lateral, and right lateral are approximately 2 : 1 : 1. The total recorded heartbeats are 27 961.

### 2.3. Data Preprocessing

BCG is generated by cardiac ejection. However, BCG recorded in a noncontact manner is mixed with respiratory effort and artifact motion. Inevitably, these components result in baseline drift and low-frequency noise, which deteriorate the performance of heartbeat detection. Therefore, prior to feeding the recorded vital signs into the developed DL model, data preprocessing is required to remove the interference of respiratory effort and artifact motion. To reduce the computational complexity, the recorded vital signs are downsampled from 1 KHz to 100 Hz, and then, a third-order Butterworth bandpass filter with bandpass frequencies of 1–7 Hz is applied [9] to remove the noise from BCG.  Figure 4 shows the vital signs before and after preprocessing. Clearly, it can be seen obviously from Figure 4 the morphology of BCG after data preprocessing.

### 2.4. Multiscale Signal Segmentation and Labeling

Unlike the existing schemes [20, 22], it is noted from Figure 4(b) that the rhythm feature of the BCG signal (J-peaks and the neighboring peaks across multiple BCGs in a large time scale), in addition to the morphological features within a single BCG duration (a relatively small time scale), can improve the ability of feature extraction, which is a benefit to heartbeat detection. Therefore, this paper proposes to take different time-scale segmentations of BCG signals as the input to enjoy the complementary advantages of both fine-grained morphological features and rhythm features. This is different from the previous DL-aided studies [20, 22]. To be specific, we divide the BCG after preprocessing into two different time segments, as shown in Figure 5. The large time-scale segment covers multiple BCG signals, while the small time-scale segment covers one BCG signal, which is located at the center of the large time-scale segment.

In general, the dominant components of one BCG signal include the H-I-J-K-L complex, ranging from 0.3 s to 1.0 s (corresponds to the upper and lower bound of heart rate 30 bpm to 120 bpm, respectively). Inspired by this fact, for the extraction of different time-scale input segments, all peaks of one selected BCG signal are considered as the candidate J-peak locations (possible heartbeat locations). For labeling, a data segment centered at every peak with the radius of *τ*_1_ samples (2 *τ*_1_ +1 samples for each segment, where *τ*_1_ covers several heartbeat intervals) is intercepted as a large time-scale segment (data segment 1), in which the one of the J-peak located at the center is labeled as “1,” and the others are “0.” Similarly, another data segment centered at the corresponding peak with the radius of *τ*_2_ samples (2 *τ*_2_ +1 samples for each segment) is intercepted as a small time-scale segment (data segment 2), and we label the segmentation of the J-peak located at the center as “1” and others as “0.” An example of data segmentation and labeling in both large and small time scales (data segment 1 and data segment 2) is shown in Figure 5.

Prior to feeding the labeled input into the deep neural network, *Z*-score normalization is applied to each BCG input segment [24] as

(1) $$\begin{array}{c} \tau^{*}=\frac{\tau -\mu }{\sigma }, \end{array}$$

where *τ* is the input segment of BCG (the lengths for large and small time-scale segment (segments 1 and 2) are 2 *τ*_1_ +1 and 2 *τ*_2_ +1, respectively) and *μ* and *σ* are the mean and standard deviation of segment *τ*, respectively.

### 2.5. ResNet-BiLSTM Deep Learning Model

Since the BCG signal contains diverse beats, which are regarded as different sequence patterns, the identification of the J-peak is challenging in practice. In this paper, a DL model combining ResNet-34 and bidirectional LSTM, referred to as ResNet-BiLSTM, is developed, where the structure of this model is shown in Figure 6. The motivation of using Bi-LSTM is to extract the high-level semantic features of time-series BCG signals as well as the memory information characterizing the dependency of features in a relatively wide time scale.

In the direction of the large time-scale segment, ResNet-34 is applied to characterize the rhythm features over multiple BCG signals. In general, ResNet-34 network is a convolutional neural network with 34 layers and contains four residual neural network units, each containing multiple convolution and pooling layers and a “shortcut connection” block. It should be noted that the H-I-J complex of the BCG signal, in comparison with the QRS complex of the ECG signal, is not obvious in the frequency domain. Thus, the convolution kernel and other parameters in the model are adjusted to accommodate one-dimensional signal input. From the model structure as shown in Figure 6, the large time-scale segment is fed into the ResNet-34 network, in order to extract the spatial characteristics, especially the rhythm features of BCG segments, over multiple heartbeat intervals. The output unit is a 512 × 16 feature matrix. In addition to the ResNet-34 model, a BiLSTM model is used to memorize the context of the input time signal, which is added to extract the temporal dependence of feature sequences extracted from BCG by ResNet-34. The output of the BiLSTM is a 128 × 1 feature vector. LSTM layers are summed into a locally focused global feature vector (containing 128 elements), which encapsulates features from the context of the current step in both forward and backward directions.

In the direction of the small time-scale segment, the single heartbeat waveform of the BCG signal also has abundant feature information, so the small time-scale segment and LSTM output feature vectors are concatenate into a one-dimensional vector (size: 257 × 1) and then put into a fully connected (FC) network to complete the classification task.

Suppose the length of input vector *x* is a one-dimensional vector (*x* × 1), and the output after convolution is further passed through a nonlinear function. The same block (linear transformation convolution + RELU) is employed again based on (2), with the shortcut connection that the input *x* is added into the nonlinear function as shown in (3) and (4) The framework of ResNet is shown in Figure 7.

(2) $$\begin{array}{c} x_{2}=\text{RELU}\left(\sum \sum G_{1}x\right), \end{array}$$

(3) $$\begin{array}{c} z_{2}=\left(\sum \sum G_{2}x_{2}\right), \end{array}$$

(4) $$\begin{array}{c} y=\text{RELU}\left(z_{2}+x\right). \end{array}$$

Table 1 shows the network parameters of ResNet-34. It can be seen that four residual units have different Conv layers. The kernel size chosen for each residual unit is identical, which is the size of 1 × 3, benefiting from the fact that the ResNet structure deepens the depth of the model, enabling it to extract deeper signal spatial features for heartbeat detection.

As a kind of time-series signals, BCG signal has an association across adjacent heartbeats, namely, the rhythmic character of BCG. Thus, to compensate for the long-term dependence that ResNet cannot capture sequence data, LSTM [25] units are employed to extract the temporal dependence of feature sequences extracted from BCG by ResNet-34. We feed the features extracted from the ResNet-34 model into the BiLSTM neural network structure for further feature extraction.

BiLSTM can utilize the information from time-series signals in the past and future of a specific time frame. The spatial BCG features are put into the LSTM neural network bidirectionally, which can extract the temporal correlations of the feature vectors from ResNet-34. The proposed BiLSTM model has one layer, and each LSTM has 128 units.

In this experiment, the leave-one out cross-validation is used to train the deep learning model. All training models use binary cross-entropy loss (BCE loss) and Adam algorithm as the optimizer [26]. The learning rate is set to 0.000 3.

## 3. Results

For the validation of the proposed heartbeat detection scheme, we conduct an experiment using a total of 440 min BCG signals measured by 21 subjects. 426 min recorded signals are used for heartbeat detection, while the rest are motion artifacts. In addition, ECG signals are simultaneously recorded by BIOPAC MP160 as a reference.

### 3.1. Evaluating Metrics

The results of heartbeat detection with 21 healthy subjects are presented in Table 2. To assess the generalizability, we consider three different performance metrics [27] to evaluate the positioning algorithm.

1. Coverage, which is defined as the ratio between the number of the correctly detected BCG over that of ECG
2. *E*_abs_, which is defined as the mean absolute error of the differences between the BCG beat-to-beat interval derived from positioning algorithm and the ECG-based beat-to-beat interval directly computed by BIOPAV MP160
3. *E*_*abs*_ defined as the mean relative error of the differences between the BCG beat-to-beat interval derived from positioning algorithm and the ECG-based beat-to-beat interval directly computed by BIOPAV MP160

Furthermore, the detection accuracy is defined using the following formula:

(5) $$\begin{array}{c} \text{Accuracy}=\frac{\text{Correct}}{\text{Correct}+\text{Incorrect}}, \end{array}$$

where Correct is the number of beat-to-beat intervals computed by the proposed algorithm with an average absolute error (*E*_abs_) less than 30 ms.

### 3.2. Performance of Different Time Scales to Detection

Firstly, the impact of the time scale for features on the detection performance is analyzed. Five different large time scales of segmentation ranging from 3 s to 11 s are considered. Comparatively, the small time-scale segmentation includes 129 samples of BCG signals of 100 Hz. For comparison, a large time-scale segment with the same time scale as the small time-scale segment is considered as the model input in order to validate the contributions of the multiscale features to the performance of heartbeat detection. The numerical results in terms of Coverage, *E*_abs_, *E*_rel_, and Accuracy are shown in Table 3, where the best performance is in bold.  Figure 8 shows the performance of large time-scale segments at different time scales.

Clearly, it can be seen that the ResNet-BiLSTM enjoys both small time-scale and large time-scale features and performs better than that with only single time-scale features, which demonstrates the superiority of the proposed multiscale design.

As regards the performance of different large time-scale segmentations, it can also be observed that the fused detection with a large time scale of 5 s (generally covers 5–8 BCG intervals depending on the heart rate) performs the best among all segmentations. A possible explanation for this result is that the signal segmentation of 5 s comprised 2-3 BCGs neighboring the signal of interest, which can benefit to characterize the rhythm features from the surrounding highly correlated heartbeats. Comparatively, the time scale of 3 s is not enough for the extraction of rhythm features, while a longer time scale >7 s introduces too much irrelevant rhythm information, resulting in feature redundancy and overfitting.

### 3.3. Performance of Different Sleep Postures

Next, heartbeat detection of different measurement postures is evaluated.  Table 4 shows the results of three measurement postures, including supine, left lateral, and right lateral. In addition, the Bland–Altman plot between the detected heartbeat and the referenced R-R interval of ECG of different measurement postures is shown in Figure 9. It can be seen that most of BCG intervals agree with those of ECG, i.e., the differences between BCG and ECG beat-to-beat intervals are within ±10 ms. The measurement posture of supine provides the best accuracy with averaged *E*_abs_ of 7.70 ms, while that of right lateral performs the worst with averaged *E*_abs_ of 15.13 ms. The results are identical to the existing schemes [28]. In conclusion, all three different measurement postures achieve the accuracy of >96.49%, which can validate the effectiveness of the ResNet-BiLSTM model.

### 3.4. Comparison with the State of the Art

In order to further validate the effectiveness of the proposed heartbeat detection scheme, the proposed method is compared with the state-of-the-art methods [17, 18, 20]. In simulations, we consider interuser comparison, where data for training and testing were measured from different subjects. We admit that due to the difference of the acquisition device, it is hard to make a precise comparison with the previous studies, but it can be generally seen from Table 2 that the proposed DL scheme examined by 21 subjects yields the mean absolute and relative errors of 9.92 ms and 2.67 ms, respectively, which are superior to the experimental results in [17, 18, 20].

Comparatively, the conventional modeling-based heartbeat detection [17, 18] performs inferior to the proposed schemes since the detection is performed within a shift window of a fixed size, which is generally insufficient to track the heartbeat detection over a wide range of heart rates. In comparison with the deep model employing the GRU network, the proposed ResNet-BiLSTM takes the complementary advantages of both morphological features in a small time scale and rhythm features in a large time scale into account and thus performs the best among different heartbeat detection schemes.

## 4. Further Study

For the training of the deep learning model, a larger dataset can help the model fit better, which can improve the robustness of the model in heartbeat detection. Therefore, in future work, we will use more subjects and longer measured BCG signals as datasets. In particular, subjects with cardiac diseases, such as arrhythmia, will be considered to examine the generalizability of the proposed model. In addition, we will also consider preprocessing the data from more scales, such as using CEEMDAN [29] (complete ensemble empirical mode decomposition with adaptive noise) to obtain different frequency components of the signal, so as to explore whether the information contained at different scales can bring better results.

## 5. Conclusion

In this paper, we developed a deep learning model for heartbeat detection from the BCG signal. Using piezoelectric sensors for vital sign acquisition, we measured BCG signals in a noncontact manner. By taking advantages of both the morphological features within a heartbeat interval and the rhythm features over multiple BCG intervals, we proposed two different time-scale segmentation and labeling to the input of the model, and the decision of heartbeat detection was based on ResNet-34 and bidirectional LSTM, which was an effective way to locate J-peaks. For validations, 21 subjects of different measurement postures were considered, and the detected heartbeat intervals from BCG were compared with R-R intervals of ECG signals. Based on experimental results, the proposed heartbeat detection performed superior to the existing benchmarks in terms of averaged accuracy and the absolute and relative errors of the beat-to-beat interval for different measurement postures. In this work, we have shown that the deep learning model plays essential to the heartbeat detection performance, and we have demonstrated that the robustness of the DL-based methods can be enhanced by taking advantages of the multiscale, which can be used as an efficient means of daily physiological monitoring.

## Figures and Tables

**Figure 1:** Flowchart of the proposed multiscale heartbeat detection scheme.

**Figure 2:** Vital sign acquisition system.

**Figure 3:** 10 s BCG manually synchronized with ECG.

**Figure 4:** 10 s segment vital signs before and after preprocessing.

**Figure 5:** Data segmentation and labeling for different time scales.

**Figure 6:** The overall framework of the ResNet-BiLSTM model.

**Figure 7:** The structure of the residual neural network unit.

**Figure 8:** Performance of heartbeat detection with different time scales.

**Figure 9:** Bland–Altman plots for different postures. (a) Supine. (b) Left lateral. (c) Right lateral. (d) All.

**Table 1:** Network parameters of ResNet-34.

Convolution layer	Kernel size	Input size	Stride, padding
Conv1	7 × 1, 32	501 × 1, 1	1,3
Max pool1	2 × 1, 32	501 × 1, 32	2,0
Conv2	3 × 1, 64	251 × 1, 32	1,1
Max pool2	2 × 1, 64	251 × 1, 64	2,0
Residual unit1	$\left[\begin{array}{c} 3\times 1,64\\ 3\times 1,64 \end{array}\right]$ × 3	126 × 1, 64	1,1
Residual unit2	$\left[\begin{array}{c} 3\times 1,128\\ 3\times 1,128 \end{array}\right]$ × 4	126 × 1, 64	2,1
Residual unit3	$\left[\begin{array}{c} 3\times 1,256\\ 3\times 1,256 \end{array}\right]$ × 6	63 × 1, 128	2,1
Residual unit4	$\left[\begin{array}{c} 3\times 1,512\\ 3\times 1,512 \end{array}\right]$ × 3	32 × 1, 256	2,1

**Table 2:** Performance comparsion between the proposed scheme and that proposed in [17, 18, 20].

Subject	Coverage(%)				E_abs_(ms)				E_rel_(ms)			
	Proposed	[17]	[18]	[20]	Proposed	[17]	[18]	[20]	Proposed	[17]	[18]	[20]
1	98.9	98.52	93.32	97.85	5.22	2.09	26.18	7.25	2.23	1.91	15.78	3.93
2	99.91	99.21	98.65	99.08	2.78	6.4	33.47	5.24	−0.35	2.15	7.9	1.24
3	99.71	99.32	98.82	99.52	3.26	4.75	22.47	6.96	1.48	0.74	7.29	2.96
4	94.92	96.43	90.12	88.24	27.35	22.36	104.8	43.75	6.21	5.72	78.8	8.87
5	99.55	98.79	89.38	99.87	5.46	6.85	125	6.01	2.99	1.93	110.4	−1.01
6	99.68	98.86	91.62	99.51	3.92	8.14	45.06	4.28	1.54	4.73	26.31	0.91
7	99.87	98.91	93.23	99.84	2.86	3.63	44.92	3.98	1.41	−2.3	17.68	2.12
8	99.67	98.83	87.62	97.60	3.59	7.52	59.3	14.11	1.39	2	45.53	1.92
9	99.98	99.25	96.77	99.84	2.05	4.97	52.18	3.04	−0.76	2.01	36.7	−1.04
10	95.72	94.12	80.08	71.13	29.3	29.21	56.5	75.21	6.25	4.23	43.29	72.38
11	89.38	93.43	93.75	86.62	29.75	33.31	71.5	58.28	6.56	9.82	60	53.22
12	98.84	98.74	92.94	98.92	7.68	10.9	33.72	8.89	3.86	4.45	18.31	7.89
13	99.33	98.13	97.85	98.41	6.11	12.12	63.06	7.81	2.01	5.34	27.06	4.69
14	99	99.3	95.46	98.30	8.46	3.64	13.96	12.17	2.88	−0.66	4.85	3.19
15	99.85	99.8	97.54	99.13	3.43	4.73	26.46	4.96	1.85	−2.13	−2.07	1.96
16	94	99.47	87.71	79.62	37.95	4.03	11.35	62.05	8.05	3.31	−2.83	38.24
17	98.81	99.38	98.02	97.61	2	4.21	47.35	3.96	2.07	1.98	34.61	1.11
18	99.44	99.28	92.74	98.20	4.02	4.77	38.56	12.26	1.5	1.66	14.34	−9.67
19	99.06	99.12	90.52	98.29	6.59	7.78	41.17	8.98	1.93	2.34	18.3	−3.85
20	99.9	93.38	96.41	99.82	3.05	33.57	34.74	4.04	1.56	12.9	15.81	2.04
21	98.63	98.41	93.55	97.75	8	10.03	17.03	10.29	4.18	4.34	3.28	5.58
Means	98.29	98.17	93.1	96.08	9.92	10.84	46.47	17.42	2.67	3.55	27.5	7.9

**Table 3:** Influence of large time-scale segments with different lengths.

Time scale	Data segment 1(s)	Data segment 2(s)	Coverage(%)	E_abs_(ms)	E_rel_(ms)	Accuracy(%)
Small time scale	1.29	1.29	96.56	15.53	6.68	95.32
Small time scale + large time scale	3.0	1.29	97.90	12.96	4.94	97.34
	5.0	1.29	98.29	**9.92**	**2.67**	**98.16**
	7.0	1.29	**98.64**	10.33	2.94	97.90
	9.0	1.29	98.52	10.94	2.95	97.65
	11.0	1.29	98.53	10.88	3.02	97.66

**Table 4:** Performance comparison for different postures.

Posture	Supine				Leftlateral				Rightlateral			
Metrics	Time (min)	*E*_abs_ (ms)	*E*_rel_ (ms)	Accuracy (%)	Time (min)	*E*_abs_ (ms)	*E*_rel_ (ms)	Accuracy (%)	Time (min)	*E*_abs_ (ms)	*E*_rel_ (ms)	Accuracy (%)
	210	7.70	1.99	98.43	111	9.15	2.53	97.32	104	15.13	4.02	96.49

## Data Availability

The data used to support the findings of this study are available from the corresponding author upon request.
